This article has been retracted.

# Clinical Study of Influence of Continuous Nursing Intervention Combined with Comfort Nursing Intervention under Medical-Nursing Combination on Self-Care Ability and Satisfaction of Elderly Patients with Chronic Diseases

**DOI:** 10.1155/2021/1464707

**Published:** 2021-10-15

**Authors:** Tian Ma, Ying Wang, Juan Liu, Aifang Wang

**Affiliations:** ^1^Health Care Rehabilitation Ward, Jinan Municipal Hospital of Traditional Chinese Medicine, Jinan 250012, Shandong, China; ^2^Department of Nephrology, Qingdao Municipal Hospital, Qingdao 266000, Shandong, China; ^3^Department of Stomatology, People's Hospital of Lixia District of Jinan, Jinan 250013, Shandong, China

## Abstract

**Objective:**

With the constant development of medical technology, the medical-nursing combination mode targeted at elderly chronic diseases has been proposed, and based on this, the study on the nursing mode of elderly chronic diseases under the background of medical-nursing combination was conducted.

**Methods:**

Total of 100 elderly patients with chronic diseases who were admitted to our hospital from April 2019 to April 2020 were selected and divided into a control group and an experimental group by lot drawing, with 50 patients in each group. Continuous nursing was conducted to patients in the control group, and continuous nursing combined with comfort nursing was performed to patients in the experimental group, so as to compare their nursing effective rate, satisfaction with nursing, self-care ability at 6 months after nursing, quality of life (QLI) scores, and blood glucose, pressure, and lipid levels at various periods.

**Results:**

Compared with the control group, the experimental group obtained significantly improved nursing effective rate, satisfaction with nursing, Exercise of Self-Care Agency (ESCA) scale scores, QLI scores, and lower blood glucose, pressure, and lipid levels at various periods 6 months after nursing, with statistical significance (*P* all < 0.05).

**Conclusion:**

Under the context of medical-nursing combination, the continuous nursing intervention combined with comfort nursing intervention is conductive to promote the self-care ability and nursing effect of elderly patients with chronic diseases and obviously improve their quality of life and psychological state.

## 1. Introduction

Chronic diseases of old age include hypertension, diabetes, insomnia, constipation, and osteoporosis. As people get older, all organ functions are constantly declining, leading to the failure to support normal human life activities and then chronic diseases. The combination of medical and healthcare refers to the form of integrating medical technology and means with nursing technology and means in daily life, which is more applicable to the elderly population. Therefore, the application frequency of medical-nursing combination in elderly patients with chronic diseases is relatively higher [1–3]. Continuous nursing means different standard continuous nursing models for different treatment and nursing periods of patients. The treatment of elderly chronic diseases requires a long time as well as physical nursing and treatment, so it is more effective to apply continuous nursing to help patients to understand the importance of chronic disease nursing and finally achieve basic self-care ability [4–6]. However, continuous nursing is an objective nursing mode performed by the nursing personnel, which may ignore some subjective feelings and needs of patients, and patients under such nursing mode are very likely to experience some adverse emotions or feelings of discomfort. Comfort nursing, as the name implies, is a nursing model that enables the maintenance of physical and mental pleasure and reduces adverse emotions in nursing subjects [7–9]. In contrast to continuous nursing, comfort nursing cares more about patients' experience and comfort and easily ignores some objective needs. Hence, combining comfort nursing with continuous nursing is more comprehensive and of great importance in physical and mental development as well as chronic disease care. The effect of combining continuous nursing with comfort nursing under the medical-nursing integration on the self-care ability and satisfaction of elderly patients with chronic diseases was explored in this study, with the results reported as follows.

## 2. Materials and Methods

### 2.1. General Information

Total of 100 elderly patients with chronic diseases who were admitted to our hospital from April 2019 to April 2020 were selected and divided into a control group (60–85 years old) and an experimental group (61–86 years old) by lot drawing, with 50 patients in each group. No statistical significance was showed when comparing their general information including gender, age, and disease type (*P* > 0.05), as given in Table 1. The study was approved by the Hospital Ethics Committee, and all patients joined the study voluntarily and signed the informed consent.

### 2.2. Inclusion/Exclusion Criteria

#### 2.2.1. Inclusion Criteria

The inclusion criteria are as follows. The patients met the clinical manifestations of elderly chronic diseases (not specifically referring to a certain type) with insidious onset, long duration, and recovery difficulty, the patients were at least 60 years old, the patients did not suffer from acute disease recently, and the patients had no history of drug allergy and drug abuse.

#### 2.2.2. Exclusion Criteria

The exclusion criteria are as follows. There were recent large fluctuations in the patients' condition, the patients had disturbance of consciousness and could not cooperate with the study, and the patients or their family members did not agree to cooperate with this study.

### 2.3. Methods

Continuous nursing based on medical-nursing combination was performed to patients in the control group. According to the disease type and personal condition, the nursing personnel established continuous nursing plans for patients, carried out different nursing standards to patients at various periods, and kept communicating with patients, so that they could understand the meaning and function of the nursing standard at each stage and promote the compliance. After the patients left the hospital, the nursing personnel paid attention to their self-care and provided relevant guidance by telephone follow-up. For example, nursing personnel conducted training and health education and promotion to all chronic disease patients for them to understand the disease causes and nursing measures. For diabetes patients, controlling and stabling their blood glucose at various periods should be the top priority of nursing personnel, so that the blood glucose was maintained normal at all times. It could be achieved by making a low-salt and low-fat dietary structure that center on coarse grain and supplemented by refined grain, associated with proper aerobic exercises. After the patient's blood glucose was under initial control, glycosylated hemoglobin was stabilized within the safe range by regular monitoring of fasting and postprandial blood glucose. For patients with hypertension, diet was one of the most important ways to control blood pressure in addition to medication control, so their diet should be bland with a high intake of vegetables and fruits. For patients with cardiovascular and cerebrovascular diseases, nursing personnel should inform them about the cause and the relationship with various indicators, such as blood glucose, pressure, and lipid, and the patients should take drugs to resist platelet concentration and learn the self-protection measures at the onset of the disease.

Continuous nursing combined with comfort nursing based on the medical-nursing combination was conducted to patients in the experimental group. During comfort nursing, nursing personnel paid close attention to patients' emotional changes, comfort, and satisfaction, so as to enable them to feel physical and mental pleasure as far as possible [8, 10, 11]. Through daily communication, nursing personnel could understand the patients' will and wishes and help them to realize some achievable wishes with the help of their family members, thus enhancing the sense of experience.

### 2.4. Observation Indexes

The nursing effective rate, satisfaction with nursing, self-care ability at 6 months after nursing, QLI (quality of life) scores, and blood glucose, pressure and lipid levels at various periods of patients in both groups were compared.

It was considered markedly effective if the clinical manifestations of chronic disease were not aggravated, and the patients had no negative emotions and other complications; effective if the clinical manifestations of chronic disease were not aggravated obviously, and the patients had relatively stable mental state and no obvious adverse reactions; and ineffective if the the clinical manifestations were aggravated, and the patients had negative emotions and serious complications.

The maximum score of the Exercise of Self-Care Agency (ESCA) scale was 100 points, and higher scores indicated better self-care ability of the tested subject [12, 13].

The scoring items of QLI included daily activities, work, and life and interpersonal relationship, and the maximum score per item was 10 points, with higher scores indicating better quality of life and vise versa.

The normal range of fasting blood glucose was 3.9–6.1 mmol/L, and the normal postprandial blood glucose was not less than 7.9 mmol/L [14].

The blood pressure included diastolic blood pressure and systolic blood pressure, with the normal range of 60–90 mmHg and 90–130 mmHg, respectively.

The venous blood was drawn in the morning on an empty stomach (fasting for 12 h and no drinking for 8 h), and the triglycerides, total cholesterol, lipoprotein, low-density lipoprotein, and high-density lipoprotein were detected by the automatic biochemical analyzer [15–17].

### 2.5. Statistical Processing

In this study, the data processing software was SPSS20.0, the picture drawing software was GraphPad Prism 7 (GraphPad Software, San Diego, USA), items included were enumeration data and measurement data, which were examined by the *X*^2^ test and *t*-test and expressed by (*n* (%)) and ($\bar{x}$ ± *s*), respectively, and differences were considered statistically significant at *P* < 0.05.

## 3. Results

### 3.1. Comparison of Nursing Effective Rates between the Two Groups

The experimental group obtained significantly higher nursing effective rates than the control group, which was statistically significant (*X*^2^ = 12.25, *P* < 0.001), as shown in Figure 1.

### 3.2. Comparison of Satisfaction with Nursing between the Two Groups

The patient satisfaction with nursing of the experimental group was obviously higher than that of the control group, which was statistically significant (*P* < 0.05), as given in Table 2.

### 3.3. Comparison of Self-Care Ability and QLI Scores between the Two Groups

The experimental group achieved remarkably higher ESCA scores and QLI scores than the control group, which was statistically significant (*P* < 0.05), as shown in Figure 2.

### 3.4. Comparison of Blood Glucose at Various Periods before Nursing and 6 Months after Nursing between the Two Groups

Before nursing, the results of comparing the blood glucose at various periods were not statistically different (*P* > 0.05), and 6 months after nursing, the fasting blood glucose and postprandial blood glucose of the experimental group were significantly lower than those of the control group, which were statistically significant (*P* < 0.05), as given in Table 3.

### 3.5. Comparison of Blood Pressure before Nursing and 6 Months after Nursing between the Two Groups

Before nursing, the results of comparing the blood pressure were not statistically different (*P* > 0.05), and 6 months after nursing, the blood pressure of the experimental group was significantly lower than that of the control group, which was statistically significant (*P* < 0.05), as given in Table 4.

### 3.6. Comparison of Blood Lipid Levels before Nursing and 6 Months after Nursing between the Two Groups

Before nursing, the results of comparing the blood lipid levels were not statistically different (*P* > 0.05), and 6 months after nursing, the total cholesterol, lipoprotein, and low-density lipoprotein levels of the experimental group were significantly lower than that of the control group; the high-density lipoprotein level of the experimental group was significantly higher than that of the control group, which was statistically significant (*P* < 0.05), as given in Table 5.

## 4. Discussion

Many old people tend to have geriatric chronic diseases, mainly because their metabolic function, immune function, and all organ functions are gradually weakened with the increasing age [10, 18, 19]. The geriatric chronic diseases mainly include endocrine system diseases, digestive system diseases, and functional diseases, which could only be controlled and treated by improving the lifestyle and eliminating bad living habits combined with some medical means, namely, the medical-nursing combination [20–22]. In addition, certain care should be conducted in the daily life of elderly patients with chronic diseases, and for those with self-help ability, such care should be done by themselves. To achieve this goal, the patients should first understand their disease and relevant precautions. Continuous nursing and comfort nursing have different focuses and can be complementary, and patients can easily miss and ignore some problems while receiving a single model of nursing. Therefore, in the overall medical environment that places equal emphasis on the importance of treatment and nursing, this study was conducted to explore the application effect and value of combining continuous nursing and comfort nursing based on the medical-nursing combination.

The study results showed that the experimental group (combining continuous nursing with comfort nursing) achieved a significantly better nursing effect and satisfaction with nursing, indicating that the combined mode enabled the patients to experience a reasonable and comprehensive professional nursing, keep a good mood and positive emotions, and stabilize the disease. Under the integration of medical care, continuous nursing with comfort nursing are combined to ensure patients receive different levels of collaborative and continuous care in different healthcare places (such as from the hospital to the family) and the same healthcare (such as different departments in the hospital) through a series of action designs, thus establishing a good communication mode between doctors, nurses, and patients, which is conducive to adjusting the psychological state of elderly patients, enhancing the participation of patients, and playing a certain positive role in the recovery of the disease.

This study also showed that the ESCA and QLI scores of the experimental group were superior to those of the control group. In Zhang' [23] study, it was pointed out that conducting continuous nursing combined with comfort nursing intervention based on medical-nursing combination to elderly patients with chronic diseases could obviously improve their adverse emotions and promote their quality of life, which was consistent with the results of this study and fully demonstrate that this study was scientific and reliable.

The ultimate goal of elderly chronic disease care is not to cure the disease, but to change the bad lifestyle of patients and effectively reduce the disease risk factors through standardized management, collaborative, and continuous care. The health status and health function of patients with chronic diseases are maintained in a relatively satisfactory state through the aged chronic disease care, so as to achieve the final purposes of reducing medication, controlling healthcare cost and saving social health resources. The result of this study shows that the blood glucose, pressure, and lipid indexes of the experimental group were superior to those of the control group, Moreover, the patients in the experimental group maintained normal blood pressure, glucose, and lipid levels, which gradually stabilized their chronic disease indexes and then greatly improved the effect of nursing accepted by them.

To sum up, performing continuous nursing intervention combined with comfort nursing intervention based on medical-nursing combination is conductive to promote the self-care ability and nursing effect and obviously improve the quality of life and mental status of elderly patients with chronic diseases.

## Figures and Tables

**Figure 1:** Comparison of nursing effective rates between the two groups. ^*∗*^Result of comparing the nursing effective rates between the two groups is statistically significant (*X*^2^ = 12.250, *P* < 0.05).

**Figure 2:** Comparison of self-care ability and QLI scores between the two groups. ^*∗*^/^*∗∗*^ESCA/QLI scores of patients between the two groups after care are statistically significant (*t* = 3.104, *t* = 5.605, *P* all <0.05). a/c indicates that there are significant differences in ESCA/QLI scores before and after nursing care in the experimental group (*t* = 8.989, *t* = 20.134, *P* all <0.05). b/d indicates that the difference in ESCA/QLI scores of the control group before and after care is statistically significant (*t* = 6.080, *t* = 14.545, *P* all <0.001).

**Table 1:** Comparison and statistics of general information ($\bar{x}$ ± *s*).

Group		Experimental group (*n* = 50)	Control group (*n* = 50)	*X* ^2^/*t*	*P*
Gender (male/female)		29/21	30/20	0.041	0.839
Age (years)		72.79 ± 5.65	72.41 ± 5.28	0.347	0.729
Height (cm)		169.39 ± 7.03	169.58 ± 7.26	0.133	0.895
Weight (kg)		64.41 ± 4.40	65.00 ± 5.32	0.604	0.547
Smoking		36	35	0.049	0.826
Drinking		40	39	0.060	0.806
Disease type	Chronic kidney disease	6	5	0.679	0.878
	Endocrine disease	10	12		
	Respiratory disease	8	10		
	Digestive tract disease	26	23		

**Table 2:** Comparison of satisfaction with nursing between the two groups.

Group	Fully satisfied	Satisfied	Dissatisfied	Total satisfaction (%)
Experimental group (*n* = 50)	38	10	2	96.00
Control group (*n* = 50)	25	12	13	74.00
*X* ^2^				9.490
*P*				0.002

**Table 3:** Comparison of blood glucose at various periods before nursing and 6 months after nursing ($\bar{x}$ ± *s*, mmol/L).

Group	Fasting blood glucose		Postprandial blood glucose	
	Before nursing	After nursing	Before nursing	After nursing
Experimental group (*n* = 50)	7.79 ± 1.33	5.11 ± 0.70	10.09 ± 1.52	7.01 ± 0.92
Control group (*n* = 50)	7.82 ± 1.32	6.33 ± 0.81	10.11 ± 1.50	8.22 ± 0.98
*t*	0.113	8.058	0.066	6.365
*P*	0.910	<0.001	0.947	<0.001

**Table 4:** Comparison of blood pressure before nursing and 6 months after nursing between the two groups ($\bar{x}$ ± *s*, mmHg).

Group	Systolic blood pressure		Diastolic blood pressure	
	Before nursing	After nursing	Before nursing	After nursing
Experimental group (*n* = 50)	152.39 ± 10.54	122.45 ± 7.08	100.24 ± 7.25	77.76 ± 4.92
Control group (*n* = 50)	153.01 ± 10.48	135.10 ± 7.71	100.11 ± 7.50	86.00 ± 5.98
*t*	0.295	8.545	0.088	7.524
*P*	0.769	<0.001	0.930	<0.001

**Table 5:** Comparison of blood lipid levels before nursing and 6 months after nursing between the two groups ($\bar{x}$ ± *s*, mmol/L).

Group	Experimental group (*n* = 50)	Control group (*n* = 50)	*t*	*P*
Triglyceride				
Before nursing	2.38 ± 0.55	2.35 ± 0.56	0.270	0.788
After nursing	0.89 ± 0.03	1.12 ± 0.16	9.991	<0.001

Total cholesterol				
Before nursing	7.73 ± 1.29	7.75 ± 1.30	0.077	0.939
After nursing	3.51 ± 0.48	5.60 ± 1.20	11.435	<0.001

Low-density lipoprotein				
Before nursing	4.66 ± 1.00	4.59 ± 0.98	0.354	0.725
After nursing	1.75 ± 0.30	2.38 ± 0.39	9.054	<0.001

High-density lipoprotein				
Before nursing	1.42 ± 0.30	1.38 ± 0.14	0.854	0.395
After nursing	3.26 ± 0.44	2.43 ± 0.47	9.116	<0.001

## Data Availability

The data used to support the findings of this study are available from the corresponding author upon request.
